The article "Innovations and Challenges in the Development of COVID-19 Vaccines for a Safer Tomorrow" was retracted in 2025. Reasons: unreliable results or conclusions; concerns about the authorship.

# Innovations and Challenges in the Development of COVID-19 Vaccines for a Safer Tomorrow

**DOI:** 10.7759/cureus.60015

**Published:** 2024-05-10

**Authors:** Devika S Kumar, Krishna Prasanth, Ashni Bhandari, Vivek Kumar Jha, Avula Naveen, Muthu Prasanna

**Affiliations:** 1 Research, Panimalar Medical College Hospital and Research Institute, Chennai, IND; 2 Department of Community Medicine, Sree Balaji Medical College and Hospital, Chennai, IND; 3 Department of Audiology and Speech Language Pathology, Shree Guru Gobind Singh Tricentenary (SGT) University, Haryana, IND; 4 Pharmacology and Therapeutics, All India Institute Of Medical Science Bilaspur, Bilaspur, IND; 5 Pharmaceutics, Pharmaceutical Biotechnology, Surya School of Pharmacy, Surya Group of Institutions, Villupuram, IND

**Keywords:** covid-19 vaccines, nanotechnology, various strategies, spike protein challenges, mutations challenging the vaccines

## Abstract

Vaccination, a historically effective public health intervention, has shielded millions from various diseases. Lessons from severe acute respiratory syndrome coronavirus (SARS-CoV) have improved COVID-19 vaccine development. Despite mRNA vaccines' efficacy, emerging variants pose challenges, exhibiting increased transmissibility, infectivity, and severity. Developing COVID-19 vaccines has faced hurdles due to urgency, limited virus understanding, and the need for safe solutions. Genetic variability necessitates continuous vaccine adjustments and production challenges demand scaling up manufacturing with stringent quality control. This review explores SARS-CoV-2's evolution, upcoming mutations that challenge vaccines, and strategies such as structure-based, T cell-based, respiratory mucosal-based, and nanotechnology approaches for vaccine development. This review insight provides a roadmap for navigating virus evolution and improving vaccine development.

## Introduction and background

Prevention and management of infectious diseases represented a paramount obstacle to human advancement and survival, similar to the current global pandemic. By stimulating an active immune response, vaccines could reduce the susceptibility of individuals [1]. Throughout history, vaccination has been an efficient public health intervention, safeguarding millions of individuals against a wide range of maladies. Researchers designed vaccines empirically in response to lessons learnt from the influenza virus, Middle East respiratory syndrome coronavirus (MERS-CoV), and severe acute respiratory syndrome coronavirus (SARS-CoV), among other kinds of viruses [2]. This method minimized the time needed for trial and error, a critical factor considering the pressing demand for a successful SARS-CoV-2 vaccine. Various vaccine formulations were developed and evaluated for their effectiveness against coronavirus disease 2019 (COVID-19). These include vaccines containing whole DNA, live-attenuated viruses, viral vectors, inactivated viruses, subunit vaccines, and mRNA-1273 (Moderna). mRNA vaccine has garnered significant interest as an innovative breakthrough in regulating the spread of the SARS-CoV-2 virus [3]. Despite achieving substantial protective effectiveness against COVID-19 at the mRNA level, the emergence of novel variants leads to the possibility of immune evasion. Newly identified variants of concern (VOCs) have caused an increase in hospitalization, infectivity, mortality, and transmissibility [4]. Among these are Alpha (B.1.1.7), Beta (B.1.351), and Omicron (B.1.1.529) [5]. The emergence of these mutated strains presents novel obstacles in the prevention and management of COVID-19, and there have been reports of reduced protective effectiveness of current vaccines. Further understanding of the immune system is anticipated to address the widespread public apprehensions regarding the efficacy of COVID-19 vaccines, in addition to mRNA vaccines, through the development of emerging technologies. Vaccines based on circular RNA, virus vectors, and nanoparticle chimeric protein can effectively combat COVID-19 [6]. The genomic sequences of SARS-CoV-2, a positive-sense, single-stranded RNA virus, and its predecessor, SARS-CoV, exhibit a near-identical structure, sharing a 79.6% sequence identity [7]. The crown-like appearance, or corona, is notably attributed to the envelope glycoprotein spike (S). This spike protein plays a vital role in viral entry, facilitating the binding to the angiotensin-converting enzyme 2 (ACE2) receptor on host cells [8]. The worldwide prevalence of SARS-CoV-2 leads to an increased viral burden in populations, thereby increasing the likelihood of new mutations emergence [9]. SARS-CoV-2 is composed of four primary structural proteins, namely the nucleocapsid (N), envelope (E), spike (S), and membrane (M) [10]. The proteins S, E, and M are within the lipid bilayer envelope, whereas the N protein envelops the viral RNA genome (Figure 1) [11]. This study emphasizes vaccine importance against COVID-19, explores mRNA tech, variant challenges, and novel vaccine approaches for effective prevention.

The article "Innovations and Challenges in the Development of COVID-19 Vaccines for a Safer Tomorrow" was retracted in 2025. Reasons: unreliable results or conclusions; concerns about the authorship.

**Figure 1:** The arrangement of SARS-CoV-2, illustrating its primary structural proteins. Image Source: Dos Santos WG, 2021 [12]; Published with permission by authors under CC BY-NC-ND 4.0 Deed (Attribution-NonCommercial-NoDerivs 4.0 International) SARS-CoV-2: severe acute respiratory syndrome coronavirus 2

## Review

Mutations challenging the vaccines

SARS-CoV-2 Genesis and Progression

Amidst the global challenges posed by the COVID-19 pandemic, various strains of the SARS-CoV-2 virus have surfaced and disseminated globally. While these new variants are inevitable in viral evolution, most of them exhibit minimal impact on the virus's mutations [13]. Nevertheless, certain mutations may result in phenotypic changes. To streamline identification and prevent discrepancies, the WHO employed the usage of the Greek alphabet such as alpha, beta, gamma, and delta (α, β, γ, δ) to designate and monitor variants of interest (VOIs) and VOCs mutations based on their global significance [14]. Presently, WHO has identified two VOCs: Delta and Omicron and had previously acknowledged eight VOIs: Epsilon, Zeta, Eta, Theta, Iota, Kappa, Lamda, and Mu [15,16]. The distinguishing features of these newly identified variants include increased transmissibility, challenges in detection through diagnostic methods, more severe clinical manifestations, evasion of natural or vaccine-induced immunity, and reduced responsiveness to treatments. The D614G mutation is common to the seven variants Alpha, Beta, Gamma, Omicron, and Mu, Delta, and Lamda, while the N501Y mutation is shared by Alpha, Beta, Gamma, Omicron, and Mu [17,18]. Further, the B.1.1.7 (Alpha), B.1.351 (Beta), and P.1 (Gamma) variants have emerged between late 2020 and early 2021 in the UK, South Africa, and Brazil, respectively [19]. Alpha and Beta variants exhibited a 50% increase in transmission, with the Alpha variant characterized by increased mortality rates and critical care unit admissions. The effectiveness of BNT162b2, ChAdOx1 nCoV-19, and NVX-CoV2373 vaccines after two doses was 93.7% against the Alpha variant [20]. For the Beta variant, the BNT162b2 vaccine provides significant protection [21]. The Gamma variant demonstrates reduced susceptibility to treatments with bamlanivimab and etesevimab monoclonal antibodies [22]. The Delta variety, first discovered in India in late 2020 has spread rapidly and is more transmissible, especially in indoor sporting environments and families [23]. The Delta variant exhibited a reduced efficacy of 33% with a single dose of Pfizer and AstraZeneca vaccines [24]. The protective effectiveness of the BNT162b2 immunization is compromised even with two doses [25]. In contrast to the Alpha variant, the efficacy of BNT162b2 two doses of vaccinations has experienced a notable decrease [26]. Lamda and Mu are currently designated as VOIs by the WHO [27]. The Lamda variant originated in Peru and Chile in late 2020, and contained the spike protein's L452Q mutation in the receptor-binding domain (RBD). Contemporary variants like Iota, Epsilon, Delta, and Kappa also share the L452R mutation [28]. The Mu variant identified in Colombia in January 2021 introduces additional intricacies to developing COVID-19 vaccines. Through emergency use authorization (EUA), COVID-19 vaccines are classified into four categories: inactivated, viral vector, nucleic acid, and subunit vaccines [29]. These vaccines are designed based on the spike protein of the SARS-CoV-2 virus, inducing the production of neutralizing antibodies and targeting the S protein to counteract viral invasion. The advent of mutations in SARS-CoV-2 presents obstacles, resulting in increased transmission, greater infection severity, diminished efficacy of antibody neutralization, and the ability to evade the immune response elicited by COVID-19 vaccines.

The article "Innovations and Challenges in the Development of COVID-19 Vaccines for a Safer Tomorrow" was retracted in 2025. Reasons: unreliable results or conclusions; concerns about the authorship.

Spike Protein Challenges

The transmembrane spike glycoprotein of the COVID-19 virus consists of two subunits: S1, which covers the surface ectodomain, and S2 for host fusion. Within the S1 subunit, the RBD facilitates viral attachment by interacting with ACE2, while the S2 subunit supports the fusion of host and viral cell membranes [30]. Consequently, the S protein has become the primary focus of antigenic interest. Concerns have been raised about the rising prevalence of genetic mutations in the viral spike protein, potentially leading to a resurgence of the virus or the emergence of a new pandemic. Specific modifications, such as D614G and N501Y, can enhance the binding affinity of SARS-CoV-2 variants to the ACE2 receptor, thereby increasing their infectivity [31]. The Delta and Omicron variants prevailed worldwide and featured a minimum of 32 mutations in the spike protein. The Omicron-form SARS-CoV-2 neutralizing antibodies (nAbs) constituted the majority of existing nAbs [32]. Given these substantial alterations, a more infectious variety than any previous VOC may arise in the near future. Interdisciplinary collaboration and a thorough scientific knowledge of the emergent "X variant" are critical. The variances between administered vaccinations and the strains currently circulating, as seen in traditional formulations like inactivated vaccines, offer minimal cross-protection. The obvious need for new vaccination technology highlights the need to address the changing scenario (Figure 2).

**Figure 2:** Spike protein challenges Image credit: Prof. Muthu Prasanna (corresponding author)

Omicron Variant Challenge

The Omicron variant affected those who had their primary vaccination series, received supplemental doses to increase immunity, and those who contracted the disease before or after vaccination [33]. The ongoing evaluation of these methods' effectiveness in reducing mortality and severe illness rates suggests resilience against initial challenges. During the sixth and seventh waves, there was a simultaneous increase in infections among those aged 60 and older, which mirrored the patterns observed in the initial waves. This trend disproportionately impacts the elderly and vulnerable populations in healthcare and community settings. The exponential proliferation of successive variants, characterized by substantial mutations (e.g., Omicron variants containing more than 50 mutations in their spike protein), requires re-evaluating the vaccination strategy [34]. The main catalyst for this transition is the declining efficacy of conventional vaccines in combating infections induced by evolving variants. As a result, consistent supplement dosages are progressively more important to preserve adequate levels of neutralizing antibodies, thereby preventing recurrent infections [35]. It is particularly hazardous to re-administer vaccines originally developed for the initial strain in a nation with higher immunization and re-infection rates. In light of this accumulated knowledge regarding mRNA vaccines, their effective manufacturing process (which incorporates adjustments for emerging variants), limited safety implications, and a strong pharmacovigilance system backed by vaccine expert committees, is advisable to adopt a dual approach. This methodology entails a primary immunization, succeeded by subsequent revaccination utilizing an alternative vaccine formulated to elicit an immune reaction against both the initial strain of SARS-CoV-2 and the most recent mutated strains. This approach guarantees all-encompassing protection against potential novel hazards [36]. As such, the European Medicines Agency (EMA) is assessing the Spanish Hipra vaccine for its capacity as a COVID-19 booster [37]. To enhance the immune response, the vaccine utilizes a recombinant protein, that mimics the RBD of the S protein in conjunction with an adjuvant. This RBD is found in both the Alpha and Beta variants of SARS-CoV-2.

The article "Innovations and Challenges in the Development of COVID-19 Vaccines for a Safer Tomorrow" was retracted in 2025. Reasons: unreliable results or conclusions; concerns about the authorship.

Various strategies

When designing vaccines based on structural guidance, the metastable prefusion conformation is chosen as the functional state for spike proteins [38]. This prefusion state must be stabilized for neutralization-sensitive epitopes to remain intact. T-cell-centered vaccinations are critical for COVID-19 immunity and long-term protection against SARS-CoV-2, specifically when circulating antibodies have a short half-life, small size, or potency [39]. Delivery to the mucosal surfaces of the respiratory system is aimed at inducing immune responses involving mucosal IgA and T cells in the respiratory tract [40]. The presentation of antigens through nanotechnologies in a multivalent approach specifically amplifies B-cell responses, potentially extending immunity duration compared to monovalent antigens [41]. Ongoing efforts are dedicated to formulate therapeutic and prophylactic measures and to address current and potential future coronavirus infections. Particular antiviral therapies do not exist for SARS-CoV-2; hence, only symptomatic treatment is currently available. Combining artificial intelligence and computational technologies is critical for accelerating medication advancement and research against this emerging disease [42]. Several medications repurposing based therapy techniques are envisaged for the prompt treatment of infected people, drawing on current genomic knowledge and protein structure modelling. Identification of targets that inhibit viral pathogenesis is essential to this advancement. One potential method uses nAbs to target the SARS-CoV-2 surface S protein. Various classic and modern lead screening methods and laboratory and animal testing are being investigated to speed up this usually lengthy and difficult procedure [43].

Structure-Based Strategy

The development of vaccination strategies has been profoundly impacted by structural biology, specifically about the SARS-CoV-2 spike protein. The S protein of SARS-CoV-2 is the main target for nAbs. The S protein trimer is anchored in the virion membrane in its prefusion (preS) form. The preS protein has been stabilized by introducing two or six proline substitutions, to generate stabilized, soluble 2P or HexaPro (6P) preS proteins. The selection of protein is predicated on the homogeneity and stability of its antigen. The proline mutation significantly impacts vaccine manufacturing, while the S-2P technique aids in quickly determining cryo-electron microscopy (cryo-EM) [44]. Vaccine design and development, including the creation of mRNA vaccines, have been expedited by this knowledge; positive results have been observed with the proliferation of advantageous proline substitutions [45]. Hexa Pro, surpass the S-2P construct in yield and stability, representing a potential breakthrough in antigen design, with multiple vaccine currently developing [46]. Beyond proline mutation, the Trimer-Tag enables the preservation of trimeric spike proteins in their native-like prefusion state. Through the incorporation of the human C-propeptide of α1(I) collagen (Trimer-Tag) into the C-terminus ectodomain of the wild-type SARS-CoV-2 S protein, the S-Trimer vaccine was synthesized [47]. The integration process results in forming a homotrimer held together by disulfide bonds. The S-Trimer maintains crucial antigenic epitopes necessary for viral neutralization, indicating the presence of a universal stabilizing mechanism that may extend to other trimeric antigens. Alum has displayed significant efficacy against circulating SARS-CoV-2 viruses, particularly the delta variant [48]. The RBM, a vital site for nAbs, is exposed in the crystal structure of the RBD-dimer, with ACE2 directly interacting with the RBM [49]. This study's findings further supported the idea that structure-based design is advantageous, as the tandem repeat single-chain dimer has the potential for enhanced vaccination effectiveness compared to the conventional monomeric variant. Various dimer forms, such as the disulfide-linked dimer and the interferon (IFN)-armed dimer, have been developed as vaccines and have demonstrated efficacy and safety against viruses [50].

The article "Innovations and Challenges in the Development of COVID-19 Vaccines for a Safer Tomorrow" was retracted in 2025. Reasons: unreliable results or conclusions; concerns about the authorship.

T Cell-Based Strategy

T-cell responses cross-react, especially those originating from tissue-resident memory T cells in the respiratory tract, hold potential as a basis for heterologous immunity against respiratory infections. The significance of T-cell-mediated immune responses has been emphasized in the creation of effective vaccines against SARS-CoV-2 [51]. In tumour immunotherapy, computational methods have been used to identify T-cell epitopes, offering precise guidance for antigen selection [52]. These epitopes pinpoint specialized algorithms and are subsequently verified through experimental confirmation. Research endeavors have concentrated on pinpointing cytotoxic T lymphocyte (CTLs) epitopes with limited mutations across individuals with diverse HLA alleles while characterizing the SARS-CoV-2 proteome. Despite these strides, the effectiveness of T-cell-based immunity in viral control remains restricted. The interplay between nAbs and T-cell immune responses, the adequacy of T-cell response magnitude for sustained efficacy, and strategies for enhancing the T-cell repertoire are still largely unexplored. CD4+ and CD8+ T lymphocytes are pivotal in managing viral infections by producing effective cytokines such as IFNγ and tumor necrosis factor (TNF) and exerting cytotoxic activities against infected cells [53]. T cells offer protection during COVID-19, particularly when the humoral immune response proves insufficient [54]. The potential drawbacks of SARS-CoV-2 nAbs generated through infection or vaccination stem from the titer decline over time and the emergence of viral escape variants [55]. Despite variations in the kinetics of nAb titers among COVID-19 convalescents, more than half experienced declining levels of nAbs after six months [56]. Sera from individuals recovering from COVID-19 and those vaccinated exhibited significantly diminished neutralizing activity against the SARS-CoV-2 Beta (B.1.351) and Delta (B.1.617.2) variants [57]. The rapid global prevalence of the Delta variant, along with the introduction of the Lamda variant (C.37), serves as a reminder that VOCs are likely to evolve persistently, presenting challenges to current vaccines heavily reliant on humoral immune responses [58].

The article "Innovations and Challenges in the Development of COVID-19 Vaccines for a Safer Tomorrow" was retracted in 2025. Reasons: unreliable results or conclusions; concerns about the authorship.

Respiratory Mucosal-Based Strategy

It has been demonstrated that intramuscular (IM) administration of COVID-19 vaccines reduces disease severity, infection, and transmission; however, they fail to effectively induce a neutralizing IgA antibody titer in the upper respiratory tract. By primarily neutralizing IgA secretion, intranasally (IN) administered mucosal vaccines can induce a more rapid and potent local antiviral immune response in the mucosa of the upper and lower respiratory tract [59]. Promoting mucosal protective immunity offers a chance to hinder virus replication and diminish their clearance through the respiratory tract mucosa. Inhaled IN mucosal vaccines possess considerable promise in preventing highly transmissible respiratory viral illnesses, including, but not limited to measles, influenza, and COVID-19 [60]. In contrast to conventional parenteral immunization, mucosal immunization offers pathogens, that penetrate through mucosal initial sites of the entrance, an active zone of defenses. Mucosal immunogenicity has the potential to elicit trained immunity, wherein innate immune cells retain an epigenetic memory of inflammatory pathogenic encounters. This memory enhances the responsiveness of the innate immune system to subsequent viral stimuli [61]. Trained immunity functions as an immediate response, which enhances the host's defensive reactions and facilitates subsequent adaptive mechanisms. The route of vaccine administration has a significant induced local immunity. For historical and emerging SARS-CoV-2 variants, intranasal vaccination provides long-lasting protection in the upper and lower respiratory tracts [62]. Current COVID-19 vaccines often fail to stimulate sufficient upper respiratory tract mucosal immunity, leading to transmission and breakthrough infections. MV130, a mucosal immunotherapy using heat-inactivated bacteria, shows promise in enhancing mucosal immunity and vaccine efficacy, offering potential solutions to these limitations [63]. MV130, a mucosal immunotherapy based on whole heat-inactivated bacteria, provides heterologous protection against SARS-CoV-2 infection in susceptible K18-hACE2 mice and improves the immunogenicity of two different COVID-19 vaccine formulations targeting the SARS-CoV-2 spike protein in C57BL/6 mice. This bacterial mucosal immunotherapy enhances the immunogenicity of COVID-19 vaccines [64]. This inactivated polybacterial mucosal vaccine, provides long-term protection against viral respiratory infections in mice through modulating the lung immune landscape. It also induces reprogramming of mouse bone marrow progenitor cells and human monocytes, promoting enhanced cytokine production. This mechanism is associated with the induction of trained immunity [65]. MV130 contains numerous cross-reactive T and B cell epitopes with high population protection coverage and potentially neutralizing B cell epitopes recognizing hemagglutinin and matrix protein 2. These results contribute to the immune-enhancing properties of MV130 observed in the clinic against respiratory viral infections [66].

The article "Innovations and Challenges in the Development of COVID-19 Vaccines for a Safer Tomorrow" was retracted in 2025. Reasons: unreliable results or conclusions; concerns about the authorship.

Nanotechnology

Vaccine carriers are currently under development, employing nanomedicine strategies. Despite this progress, there was limited exploration of alternative nanotechnology approaches to address the ongoing COVID-19 pandemic. Nanocarriers play a pivotal role in managing the pharmacokinetics and pharmacodynamics of antiviral drugs, overcoming challenges like limited bioavailability and inadequate solubility. Consequently, these factors contribute to prolonged virus suppression, reduced toxicity, improved drug bioavailability, and lower dosage requirements [67]. Actively targeted nanocarriers have demonstrated the ability to overcome biological barriers, from delivering therapeutic concentrations to protected viral reservoirs [68]. Nanocarriers also play a crucial role in neutralizing biological agents such as antibodies, proteins, peptides, and RNA interference, significantly enhancing the therapeutic management of COVID-19 [69]. Key advantages of vaccine nanocarriers lie in their nano size, aligning with the nano size of many biological systems such as viruses (including SARS-CoV-2) and proteins [70]. By surpassing tissue barriers and precisely targeting essential anatomical sites like lymph nodes, nanoparticles offer a significant advantage over traditional administration methods, including subcutaneous, intramuscular, mucosal, epithelial, oral, respiratory, and digestive routes [71]. Given the ongoing COVID-19 pandemic, there is substantial concern about the potential of vaccine adjuvant nanoparticles (VANs) to enhance the safety and efficacy of the immune response. Vaccine adjuvants are vital for dose-sparing, reducing the required antigen dosage, enhancing production capacity, and expanding vaccine accessibility to a broader demography. Preclinical development is underway for vaccines targeting COVID-19, utilizing five protein subunits with an adjuvant and antigen combination [72]. Clinical trials are anticipated to commence shortly for NVX-CoV2373, a recombinant SARS-CoV-2 glycoprotein-based nanoparticle vaccine with adjuvant matrix. Potential nanotechnology applications in COVID-19 therapeutics and vaccine research include stimulating immune responses and improving antigen cross-presentation to T cells [73]. Researchers must comprehensively understand pathophysiology, immunological response, and structural morphology. In conclusion, while vaccine carriers using nanomedicine strategies show promise, further exploration of alternative nanotechnology approaches for COVID-19 is crucial. Nanocarriers offer significant advantages in drug delivery, overcoming bioavailability challenges, and enhancing therapeutic management, underscoring their potential in combating the pandemic. Clinical trials, like NVX-CoV2373, exemplify nanotechnology's role in advancing COVID-19 therapeutics.

The article "Innovations and Challenges in the Development of COVID-19 Vaccines for a Safer Tomorrow" was retracted in 2025. Reasons: unreliable results or conclusions; concerns about the authorship.

Challenges

Developing a COVID-19 vaccine encountered numerous hurdles due to the urgent need, limited understanding of the virus, and the imperative need to balance speed with safety. Ensuring vaccine safety and efficacy demands meticulous testing to identify potential side effects. Striking the right balance between fast development and thorough testing was critical. The virus's genetic variability required ongoing adjustments of vaccine formulations and address emerging variants. Mass production and distribution proved challenging, necessitating the scaling up of manufacturing capabilities while maintaining stringent quality control. International collaboration emerged as a vital component, demanding coordination among governments, researchers, and pharmaceutical companies. Overcoming vaccine challenges involves addressing public concerns and disseminating accurate information. Equitable access became a global priority, aiming to prevent disparities in vaccine distribution between affluent and less privileged nations. Despite these challenges, successful vaccine development showcased the effectiveness of global cooperation and scientific innovation. However, ongoing efforts are essential to monitor long-term vaccine safety, address emerging variants, and ensure widespread access to achieve lasting control over the pandemic.

## Conclusions

The rapid progress in developing COVID-19 vaccines represents an accomplishment in medical research and public health. With unprecedented collaboration between researchers and pharmaceutical companies worldwide, safe and efficacious vaccines were created faster to combat the global pandemic triggered by the novel corona virus. These vaccines have played a pivotal role in mitigating the virus's impact and preventing severe illness, hospitalizations, and fatalities. Vaccination campaigns have significantly contributed to attain herd immunity in numerous regions, aiding in curbing the virus's spread and facilitating societies in returning to a semblance of normalcy. Despite these achievements, challenges such as vaccine distribution, hesitancy, and the emergence of new variants persist and require ongoing attention. Continuous research and surveillance are vital to adapt and enhance vaccination strategies, ensuring vaccine effectiveness against evolving virus strains is imminent. In conclusion, the development of COVID-19 vaccines exemplifies a triumph of scientific collaboration and innovation. While these vaccines are essential for managing the spread of the virus, it is crucial to maintain ongoing efforts to guarantee global accessibility, tackle emerging obstacles, and uphold vigilance in the ongoing fight against the pandemic.
